# Prevalence of stress and its determinants among residents enrolled in China Standardized Training Program for Resident Doctor (C-STRD) program: A cross-sectional study

This article has been retracted.

**DOI:** 10.1371/journal.pone.0207258

**Published:** 2019-01-07

**Authors:** Ying Jiang, Yan-Jun Guan, Da-Wei Dai, Wei Huang, Zhen-Yu Huang

**Affiliations:** 1 Department of Medicine, New Jersey Medical School Affiliated to Rutgers University, Rutgers University, Newark, New Jersey, United States; 2 Department of Neurosurgery, Shanghai Chang Zheng Hospital affiliated to China Second Military Medical University, Shanghai, PR China; Indiana University, UNITED STATES

## Abstract

**Background:**

It has been widely understood that well-trained doctors are crucial for a high-quality public health system and safe patient care. Thus, in 2011, China initiated its first national residency training program, called the *China Standardized Training for Resident Doctor* (C-STRD), for medical graduates to prepare qualified doctors for the medical care system with increasing demands. So far, no studies have specifically address the prevalence of stress and its determinants among residents enrolled in the C-STRD.

**Participants and methods:**

The research is performed in two stages. In stage I, the authors conducted a pilot study and met 112 C-STRD residents in person. Based on the preliminary data, a revised questionnaire was adopted in stage II, during which the authors conducted a multi-institutional, cross-sectional survey of 340 participants from 11 hospitals in Shanghai in a self-administered manner.

**Results:**

The results showed that C-STRD residents were overall under severe stress as their mean PSS score was 27.5 ± 4.9, which was higher than the threshold of high stress (PSS = 20). Specifically, the PSS score for the residents with Bachelor (MB), Master (MM) and Doctoral of Medicine (MD) educational degree were 26.6 ± 4.1, 27.8 ± 3.5 and 27.1 ± 5.2, respectively (P>0.05). Their stress was mainly associated with their financial income status and workload, as these two factors caused more severe burden than other listed stressors (P<0.05). Specially, the residents indicated that their montly payroll amout were as low as $590.2 ± 127 while no benefit package and allowance were given. Surprisingly, wage arrears up to 5.3 month were reported by 36 (10%) participants. Workload survey showed the residents has high work intensity and inadequate rest. Since no stress management program was provided, the majority of residents tended to cope their stress with unhealthy strategies, such as mesmerizing in TV/computer (88.2%) and overeating (59.7%).

**Conclusion:**

The C-STRD residents are at high risk of perceived stress. Although there was a difference in perception of stress for workload and career future among different educational degree owners, low financial income is the major stressor among all C-STRD residents. Unhealthy stress management strategies were adopted by all residents due to lack of appropriate stress-relieving intervention.

## Introduction

It has been widely understood that well-trained doctors are crucial for the high-quality public health system and safe patient care. For medical school graduates, residency training is a crucial stage for them to gain both knowledge and skill before they become fully professional. However, residency training is very stressful [1, 2]. Typically, residents are constrained by long working hours, high job demands, sleep deprivation and personal time inadequacy [3, 4], which had been shown to cause stress symptoms and lead to both emotional exhaustion and negative consequences on residents’ mental as well as physical well-being [5, 6]. Thus, it is important to identify specific stressors and prevent the ultimate burnout [7].

In 2011, the Health Department of China officially introduced its first nationwide residency training program for fresh medical graduates as one of many important procedures in this round of medical reform. This residency training program is known as the China Standardized Training for Resident Doctor (C-STRD) [8]. The C-STRD is mandatory and can take up to 3 years according to the educational degree of participants. All class 2011 and after are required to participate. Specifically, the training period for Doctoral (MD), Master (MM) and Bachelor (MB) degree of Medicine are one, two and three years, respectively. At the end of the training, all participants are required to take a comprehensive test to ensure their medical skills and knowledge. Once achieved the completion certificate, they are again sent back to the market and hunt for their future employer by themselves. According to original enrollment plan, 7902 medical graduates had already been enrolled into the C-STRD by 2014 [9].

So far, multipe studies had already evaluated various stressors in different residency training program throughout the world [1, 10–15]. However, we struggled to identify the prevalence of stress and specific stressors of participants enrolled in the C-STRD as no study has explored the prevalence and sources of stress among this population. Thus, the purpose of this study was to determine the stress sources and prevalence of C-STRD enrolled residents.

## Methods

### Study design and instruments

The current study has been approved by the ethics committee of Shanghai Chang Zheng Hospital. Overall, the current study was developed by the authors according to previously introduced questionnaire-development process [16, 17]. The current study was conducted in two steps.

The first step involved a pilot study to collect preliminary data for questionnaire development. First, the author performed a literature search and failed to found any readily-available instrument that was suitable for the current study. Thus, the author developed a preliminary questionnaire, which included literature-adopted and self-developed questions. To validate this self-developed questionnaire, the authors met 112 C-STRD residents in person from five general hospitals in Shanghai. The authors discussed with these residents about their life stressors and collected over 20 kinds of stressors they mentioned. The stress level caused by these stressors were discussed as well as their stress-dealing methods. By comparing the frequency of these stressors mentioned by the residents during analysis of preliminary data from the pilot study, the authors listed 7 stressors into the final formal questionnaire, which were identified as the most stressful factors by the participants from the pilot study as well as the medical students from literatures [13, 18–22]. Furthermore, the formal questionnaire was further developed focusing on the top two stressors from the pilot study.

For the final questionnaire, the demographic profiling and Perceived Stress Scale (PSS) were directly used as that from the pilot study without any revision. The standard 10-item PSS was used to understand the participants’ perceived stress related to current objective events [23]. The PSS is a self-reported instrument with ten items and each item is rated on a five-point Likert-type scale (0 = never to 4 = very often). Its threshold of high stress is defined as larger than 20 points [23]. It has been previously validated and utilized by several successful investigators researching students’ stress levels [13, 24, 25]. The current study adopted the Chinese version of the PSS without any amendment, the validation of which had been previously verified [26]. The final PSS scores came from the summary of all items and a higher score indicated greater psychological stress. Next, for the stressor fact and stress-reducing intervention study, the 7 most mentioned stressors from the pilot study were listed along with most mentioned stress-reducing interventions by the respondents and literatures [27]. Next, the questions involved in the workload and financial status were borrowed from previous studies without any amendment from the pilot study [13, 14, 18–21, 28, 29].

Then, the formal survey was conducted by using the final validated questionnaire. The entire questionnaire could be read in S1 Table. Eleven coordinators from 11 hospitals personally distributed printed-questionnaires to C-STRD participants from their designated hospitals. To ensure the maxim respond rate, the coordinators collected the completed questionnaire in person after the questionnaire was completed. Participation was voluntary, anonymous and without any incentives.

### Participants

The cross-sectional survey took place in 11 general teaching hospitals in Shanghai, China between January and September 2014. Participants were doctors participated in the C-STRD program. A paper-based questionnaire was sent to 500 current or formal C-STRD-enrolled residents and the overall respond rate was 68%. Table 1 listed the general questions dealing with the demographic data of participants. For each question in the questionnaire, the lowest respond rate is 91.2%.

**Table 1:** General information of all the C-STRD residents who participated in the survey.

	Total	Bachelor of Medicine	Master of Medicine	Doctor of Medicine
**General information**				
male	200	20	84	96
female	140	20	72	48
age	27.0 ± 8.4	24.4 ± 1.1 ^a^	27.3 ± 1.5 ^b^	29.2 ± 1.4 ^c^
**Marriage Status**				
married				
partner living together	106	0 (0%)	43 (27.6%)	63 (43.8%)
partner living separately	30	0 (0%)	17 (10.9%)	13 (9%)
divorced	2	0 (0%)	1 (0.6%)	1 (0.8%)
**Having kid(s)**				
one	56	0 (0%)	16 (10.3%)	40 (27.8%)
≥ two	3	0 (0%)	1 (0.6%)	2 (1.4%)
**Living condition**				
Shared apartment	185	25 (62.5%)	92 (60%)	68 (47.2%)
Living with parents	87	15 (37.5%)	39 (25%)	48 (33.3%)
By self or with wife	68	0 (0%)	25 (16%)	28 (19.4%)

Value was presented in the mean ± standard deviation. The earning and expenditure amount was presented in US dollar. Items marked with different English letter indicated statistical difference (P<0.05).

### Statistical analysis

The statistical analysis was performed using the GraphPad PrismTM 7.0 (GraphPad Software, San Diego, CA, USA), and descriptive statistics were performed. Data was presented as mean ± standard deviation. In the financial situation section, all income amount had been converted into US dollar with the exchange rate of 1 dollar against 6.1 China RMB. The one-way ANOVA was used to compare the difference of demographic features (Table 1), PSS score (Table 2) and financial status among participants with different educational degree. The one-way ANOVA was applied to the Total Score comparison (Table 3) while the one-way ANOVA on ranks test (a.k.a. Kruskal-Wallis test), following the post hoc test, was used to check for detailed difference of stressor fact (Table 3) and workload among participants with different educational degree. *P* value <0.05 was considered statistically significant for the entire study, except for Table 3, the significant level of the Kruskal-Wallis test was set for 0.01.

**Table 2:** Responses to the perceived stress scale from the C-STRD residents (N = 340).

Perceived stress scale	Never	Almost never	Sometimes	Fairly often	Very often	Average PSS score
How often have you been upset because of something that happened unexpectedly?	10	32	115	153	30	2.59 ± 0.27
How often have you felt that you were unable to control the important things in your life?	8	31	120	169	12	2.57 ± 0.33
How often have you felt nervous and “stressed”?	5	29	80	78	148	3.35 ± 0.65
In the last month, how often have you felt confident about your ability to handle your personal problems?	50	137	115	30	8	2.62 ± 0.28
How often have you felt that things were going your way?	31	162	132	11	4	2.64 ± 0.25
How often have you found that you could not cope with all the things that you had to do?	14	13	151	142	20	2.4 ± 021
In the last month, how often have you been able to control irritations in your life?	35	154	127	18	6	2.62 ± 0.26
How often have you felt that you were on top of things?	63	161	106	6	4	2.84 ± 0.26
How often have you been angered because of things that were outside of your control?	7	23	74	157	79	2.92 ± 0.27
How often have you felt difficulties were piling up so high that you could not overcome them?	2	37	97	200	4	2.67 ± 0.38

The numbers listed in the table indicated how many participants selected the specific item.

**Table 3:** The C-STRD residents’ stressor fact.

Stressor	Total	MB	MM	MD
**Can you rate the following stressors in a 0 to 10 range?** ***				
Financial income	9.2 ± 0.7 ^a^	9 ± 1.4	9.1 ± 1.1	9.4 ± 0.9
Workload	7.4 ± 1.3 ^b^	5.7 ± 2.1	7.4 ± 2.1	7.8 ± 1.3
Unclear long-term career future	6.9 ± 1.4 ^c^	6.3 ± 2.3	6.9 ± 2.1	6.9 ± 1.8
Supporting family	6.5 ± 1.2 ^c^	5.4 ± 1.9	6.5 ± 1.7	6.9 ± 1.8
Job environment (dealing with patients)	6.4 ± 1.3 ^c^	5.4 ± 2.2	5.9 ± 1.9	7.1 ± 1.9
Relationships with trainers	3.7 ± 1.3 ^d^	5.7 ± 2.2	3.3 ± 1.7	3.6 ± 1.9
Relationships with colleagues	3 ± 1.4 ^d^	3.1 ± 2.1	3.4 ± 2.1	2.7 ± 2.1
**How do you dealing with your stressors?** ^###^				
Mesmerized in front of TV or computer	300 (88.2%) ^a^	39 (97.5%)	136 (87.2%)	125 (86.8%)
Overeating	203 (59.7%) ^b^	28 (70.0%)	75 (48.1%)	100 (69.4%)
Drinking & smoking	176 (51.8%) ^b^	20 (62.5%)	80 (51.3%)	71 (49.3%)
Talk to colleagues	98 (28.8%) ^c^	15 (37.5%)	54 (34.6%)	29 (20.1%)
Talk to family	60 (17.6%) ^c^	24 (60.0%)	19 (12.2%)	17 (11.8%)
Self-mutilation	9 (2.6%) ^d^	5 (12.5%)	2(1.3%)	2 (1.4%)
Talk to trainers	4 (1.2%) ^d^	0 (0%)	4 (2.6%)	0 (0%)
Stress management	0 (0%) ^d^	0 (0%)	0 (0%)	0 (0%)
Other method	0 (0%) ^d^	0 (0%)	0 (0%)	0 (0%)
**Have you ever had thoughts of quitting medical profession? (answered yes)**	225 (66.2%)	21 (52.5%)	100 (64.1%)	104 (72.2%)

Each value was presented in the mean ± standard deviation. The one-way ANOVA was applied to the Total Score comparison (comparison was made in the same column). Items marked with different English letter indicated statistical difference among all stressors and methods dealing with stressors (P<0.05). Then, the one-way ANOVA on ranks test (a.k.a. Kruskal-Wallis test), following the *post hoc* test, was used to check for detailed difference among participants with different educational degree (comparison was made in the same row). Items marked with wavy line indicated statistical difference among different educational degree (P<0.01).

*** Self-evaluated in a 0 (poor/none) to 10 (excellent/tremendous amount) scale.

^###^ The numbers listed outside the parentheses indicated how many participants selected the specific item while the numbers inside the parentheses indicated the corresponding percentage.

## Result

### Demographic profiles

Table 1 listed the socio-demographic characteristics of the C-STRD residents participated in the survey. Overall, the majority [200 (58.8%)] of the respondents were male and aged 28.3 ± 2.1 on average while that of the female [240 (41.2%)] were 26.9 ± 1.8. Of those that responded, 144 (42.4%), 156 (45.9%) and 40 (11.8%) had MD (Doctoral degree of Medicine), MM (Master degree of Medicine) and MB (Bachelor degree of Medicine), respectively. At the time of the survey, the majority of the participants [136 (40%)] were married, 59 had kid(s) (17.3%) and 185 lived in a shared apartment (54.4%).

### Perception of the stress

Next, the PSS was used to measure the recent perception of the stress of the participants in Table 2. All residents scored 27.3 ± 4.9 on average (ranged from 11 to 40). Specifically, the PSS score for the MB, MM, and MD residents were 26.6 ± 4.1, 27.8 ± 3.5 and 27.1 ± 5.2, respectively, and no significant difference was observed among them (P>0.05). The top three causes resulted in this constant stress were that the participants “very often felt nervous and stressed” (PSS score 3.35 ± 0.65), their “things were very often out of control” (2.92 ± 0.27) and “they were never on top of things” (2.84 ± 0.26).

### Key stressors identification and coping strategies

Table 3 listed stressors fact reported by the residents. Overall, the top three stressors included their financial income status (stress level = 9.6 ± 0.4 in a 0–10 scale), workload (stress level = 7.2 ± 2.1), and unclear long-term career planning (stress level = 6.6 ± 1.8). Statistical analysis indicated that financial income and workload caused significantly higher stress level than other listed stressors (P<0.05). Additionally, compared to the MB residents, the MM and MD suffered significant higher stress level due to heavy workload and family supporting (P<0.05). However, the MB residents had more tense relationships with trainers than that of the MM and MD (P<0.05). To deal with their stress, the majority of residents [300 (88.2%), P<0.05] selected to mesmerize themselves in front of TV or video game as their prime choice, which was followed by the choice of overeating [203 (59.7%)] and drinking/smoking [176 (51.8%)]. Surprisingly, 9 participants (2.6%) picked to harming self rather than talk to their family, trainers or colleagues. We also found that none of the residents (0%) went for stress management because they had never been provided with such service from their training hospital and C-STRD program. Under such stress, 225 participants (66.2%) had generated the thoughts of quitting medical profession, which was highest among the MD residents (P<0.05).

### Contributing factors of the key stressors

Table 4 showed the detailed fact of C-STRD residents’ financial status. The average monthly payroll amount was $632 ± 414.1 according to all respondents. Specifically, this amount was $590.2 ± 127, $604.9 ± 200.4 and $702 ± 186 for the MB, MM and MD, respectively (P<0.05). There was no benefits package provided and no allowance for overtime working. Surprisingly, 9 participants (10.6%) also reported wage arrears, and the longest of arrear period was 5.3 month by the time of the survey. Contrary to their low income, the expenditure of participants were tremendous. The home mortgage, apartment rent, family provision, transportation fee and food were ranked the top 5 major expenditures.

**Table 4:** The C-STRD participants’ financial status.

Financial status	Total	MB	MM	MD
**What is your income situation?**				
Monthly payroll Amount	632 ± 414.1	590.2 ± 127 ^a^	604.9 ± 200.4 ^b^	702 ± 186 ^c^
Benefit package	no			
Allowance (including for overtime-work)	0			
Wage arrears	Reported by 36 respondents (10.6%) (the longest period was 5.3 months at the time of survey)			
**What is your major living cost? (% relative to payroll)**	ranking			
Monthly home mortgage	1	0 (0%)	852.5 ± 480 (141%)	1271.6 ± 164.9 (181%)
Monthly apartment rent	2	186.9 ± 48.4 (32%)	384.1 ± 233.3 (63.5%)	400.2 ± 172.0 (57%)
Family provision	3	0 (0%)	149.9 ± 58.3 (25.4%)	153.3 ± 30.5 (25.3%)
Food	4	104.9 ± 89.1 (17.8%)	123.3 ± 49.5 (20.4%)	133.8 ± 49.9 (19.1%)
Transportation	5	59.5 ± 36.4 (10.1%)	62.3 ± 35.9 (10.3%)	58.9 ± 23.9 (8.4%)

Each value was presented in the mean ± standard deviation. The one-way ANOVA test was used to compare the monthly payroll amount among residents with different educational degree. The payroll amount had been converted into US dollar with the exchange rate of 1 dollar against 6.1 China RMB. Items marked with different English letter indicated statistical difference (P<0.05).

Table 5 demonstrated the details of resident’s workload. All residents evaluated their work intensity as 9.2 ± 1.5 and 6.6 ± 2.4 out of 10 on weekdays and weekends, respectively. Specifically, they served the 24 hrs on-call shift every 4.7 ± 1.7 days. During weekdays, the residents need to see 31 ± 6.7 patients/month, conducted 7.1 ± 2.4 surgeries/week for surgical residents and worked overtime 12.8 ± 10.7 hrs/weekdays while only had 1.6 ± 1.4 hrs/day for a break. Meanwhile, 261 participants (76.8%) worked overtime in the hospital for 7.5 ± 7.1 hrs during the weekend. Additionally, 146 participants (42.9%) also conducted lab research after work for 5.1 ± 2.7 hrs/week while 70 participants (20.6%) performed non-educational for 2.3 ± 3.4 outside the hospital. The majority of these non-educational activities included being messengers, preparing lecture notes for the trainer, delivering packages, and even helping trainer with house moving. Under such intensive workload, most of the residents [265 (77.9%)] could only sleep 4 to 7 hrs a day and 69.1% reported they remained unrefreshed after sleep. Detailed comparison among residents with different educational degrees could be reviewed in Table 5.

**Table 5:** The C-STRD participants’ working fact.

Workload survey	Total	MB	MM	MD
**Can you provide the following factors during (9 hrs) normal working?**				
Working intensity index*	9.2 ± 1.5	9.2 ± 1.3	9.0 ± 1.4	9.4 ± 1.1
On-call cycle (days)	4.7 ± 1.7	4.6 ± 1.4	5.1 ± 1.1	4.5 ± 1.1
Managing life-threatening situation (answered yes)	316 (92.9%)	35 (87.5%) ^a^	141 (90.3%) ^a^	140 (97.2%) ^b^
Duration of break time per day (hrs)	1.6 ± 1.4	1.5 ± 0.9	1.4 ± 1.1	1.9 ± 1.0
Number of inpatients seen in wards per month	31 ± 6.7	30.6 ± 5.6	31.5 ± 6.4	30.9 ± 5.1
Number of surgeries per week (for residents of surgery department)	7.1 ± 2.4	6.6 ± 2.1	7.1 ± 1.9	7.7 ± 1.4
**Can you provide the following factors during your overtime working period?**				
Working intensity index*	6.6 ± 2.4	7.4 ± 2.1 ^a^	6.0 ± 1.6 ^b^	6.4 ± 1.1 ^b^
Overtime on weekdays (answered yes)	340 (100%)	40 (100%)	156 (100%)	144 (100%)
Entire overtime hours per weekdays	12.8 ± 10.7	12.9 ± 4.6	13.5 ± 9.7	11.9 ± 7.1
Overtime on weekend (answered yes)	261 (76.8%)	31 (77.5%) ^a^	110 (70.5%) ^b^	120 (83.3%) ^c^
Entire overtime hours per weekend	7.5 ± 7.1	8.7 ± 3.8 ^a^	7.6 ± 6.4 ^b^	6.1 ± 2.5 ^c^
**Do you need to participate in lab research?**				
answered yes	146 (42.9%)	7 (17.5%) ^a^	85 (54.5%) ^b^	54 (37.5%) ^c^
Lab research time (hours/week)	5.1 ± 2.7	5.1 ± 1.8	4.8 ± 2.5	5.2 ± 1.9
**Do you need to participate in non-educational activities?**				
answered yes	70 (20.6%)	11 (27.5%) ^a^	35 (22.4%) ^ab^	24 (16.7%) ^b^
Non-educational activities time (hours/week)	2.3 ± 3.4	3.1 ± 2.8 ^a^	1.8 ± 2 ^b^	2.1 ± 2.7 ^b^
**How long does your sleeping last?**				
< 4 hrs	58 (17.1%)	7 (17.5%) ^ab^	21 (13.5%) ^a^	30 (20%) ^b^
4–7 hrs	265 (77.9%)	24 (60%) ^a^	134 (85.9%) ^b^	107 (74.3%) ^c^
≥ 7 hrs	17 (5%)	9 (22.5%) ^a^	1 (0.6%) ^b^	7 (4.9%) b
Report to feel refreshed after sleeping? (answered yes)	105 (30.9%)	20 (50%) ^a^	37 (23.7%) ^b^	48 (33.3%) ^c^

Each value was presented in the mean ± standard deviation. The one-way ANOVA on ranks test (a.k.a. Kruskal-Wallis test), following the *post hoc* test, was used to check for detailed workload difference among participants with different educational degree (comparison was made in the same row). Items marked with different English letter indicated statistical difference (P<0.05).

* Self-evaluated in a 0 (poor/none) to 10 (excellent/tremendous amount) scale.

## Discussion

It has been widely understood that well-trained doctors are crucial for the high-quality public health system and safe patient care. However, during practice training, medical residents entail high prevalence of stress, which can cause mental health issues [30, 31], affect training quality, and change residents’ attitude towards their future career [10–12, 32–35]. Additionally, high prevalence of stress had been not only observed in medical students from western countries [36–40], but also those from Asian regions/countries, such as Hong Kong[41], Korea [42], Malaysia[43], Thailand [44], and Saudi Arabia [45]. Unfortunately, no such study was performed in mainland China. Thus, we conducted the first comprehensive multi-institutional study focusing on the magnitude of perceived stress among C-STRD enrolled residents in China. Based on our survey, we concluded that 1) the C-STRD enrolled residents demonstrated a high level of stress, 2) although residents with different educational degree responded to various major stressors with disparity, low financial income is the major stressor among all C-STRD residents, and 3) a proper stress reduction program is in urgent need for C-STRD residents to cope with their stress.

Our core objective was to identify whether C-STRD residents are under stress and subsequently identify the sources of stress. Keeping with the tradition of maximum prudence, we utilized the PSS scale and identified that C-STRD enrolled residents scored above the threshold of high stress. Compare to other international studies, the C-STRD residents’ PSS scores were not only significantly higher than that of the societal normative populations [10, 14], but also surpassed their foreign counterparts [1, 10–14]. For residents with less extreme duty hours, the PSS score varied from 22 in 938 residents in Saudi Arabia [1] to 16.1 in 168 family medicine residents in the US [12]. On the other hand, Zaré et al. [14] showed that US general surgery residents who work for 80 hrs/week reported the PSS score of 26.8. Collectively, these data indicated C-STRD residents suffered a high level of stress.

The literature demonstrates that medical residents shoulder higher levels of debt had higher incidences of burnout [46], depressive symptoms, cynicism [47] and decreased career satisfaction [48]. Our data indicated that the C-STRD residents were majorly struggled with their low income and high expenditures for the bare necessities of life. According to the 2011 data published by the China Bureau of Statistics, the average income for the Bachelor and graduated degree owner were $720 and $1007, respectively, [49]. However, according to our survey, residents’ payroll varied from $590.2 ± 12 for the MB residents to $770.2 ± 186 for the MD residents, who were significantly underpaid compared to the national salary average. Not only had we observed a low monthly income and purchasing power, the C-STRD residents spent a large proportion of their income on life necessities as well. The majority of the C-STRD enrolled respondents lived in rented apartments, which cost as high as 63.5% of their entire income. This is not the worst as for those who had a home loan (second majority group), their income was not even enough to cover the monthly installment. These numbers were much higher than the average Shanghai household final consumption expenditure on housing/living (9%) [50]. Thus, it is reasonable to conclude that C-STRD residents are deeply concerned about their financial status. Surprisingly, the wage arrears were reported by more than 10% of all respondents, which makes the financial status even more difficult for those doctors. As more than one-third of MM and MD are married or even have kids, it is understandable that they are unsatisfied with their current income and feel life is extremely stressful for them.

Heavy workload was also reported as one the highest-ranking stressors by the C-STRD residents, which concurred with other studies [13, 14, 28, 29]. Additionally, the current study also replicated data from previous studies, which identified major parameters associated with the stronger workload in residents, such as overtime working, high patient load, critical situation management, on-call duty cycle, short break time and poor sleep quality and quantity [1, 12, 51]. Based on our calculation, the C-STRD residents spend averagely 78.5 hrs/week on duty in hospital, which is fairly close to the 80 hrs/week restriction of the US residents training program [52]. Existing literature describes that 80 hrs/week policy on patient safety and residents’ well-being are equivocal. For residents, it improves their lifestyle, sleep quality, mood, testing scores and operative case volume [14, 53, 54]. For patients, decreased errors and improved care were also monitored [55]. Thus, our data indicated that the C-STRD residents should be able to handle their current workload with no problem. However, additional to the regular “clinical requirements”, nearly half of the C-STRD residents participated in lab research for 5.1 hrs/week. Although 100% reported they worked voluntarily, more time not at home translates to less time available for personal and family pursuits. Last but not least, the C-STRD residents also conducted non-educational activities as those from other institutes [56], which could be the last straw to totally burn-out already-stressful C-STRD residents.

Our results concerning the current psychological wellbeing of C-STRD residents raised the question of appropriate intervention. Previous literature demonstrated that residents appeared to be protected from stress by some support mechanisms, such as providing support groups, professional and career counseling, psychological counseling, financial support, insurance, family and child care, and legal advisors to address malpractice [27]. Surprisingly, no C-STRD residents sought formal counseling or intervention to healthily perceive these stresses as none was provided by the current training program. It is worth mention that the mentoring program is thought to one of the most important options to providing professional and emotional support to residents. Unfortunately, we also observed the lack of communication between residents and their trainees, which is consistent with previous literature [57–59]. As problems faced by the residents remained unidentified by the trainees, residents’ stressors, therefore, remain un-addressed.

This study was subject to some limitations associated with experiment design. First, each department had varied minimum education degree requirement for participants during enrollment. The department of surgery and internal medicine required participants to obtain either MD or MM degree while the others (such as the department of radiology) required only the MB degree. Due to the nature of the surgery and internal medicine, participants in these departments should have a heavier workload than other departments, which can cause higher stress level and bias in our survey results. Additionally, literature had reported female residents tended to have higher stress level than their male counterparts [19]. However, the current study did not separate the female residents from the male due to relative small sample size issue. Thus, the difference during the original admission demographic characteristic led to unbalanced educational degree distribution and gender ratio. Additionally, the PSS is normally considered as a short-term stress measuring scale. Longer follow-up periods are needed to better understand the stress level changes and coping strategies’ outcomes. The response rate in the current study is 68%, which may introduce bias during data interpretation and analysis. Moreover, Shanghai is the largest metropolitan in China, which has its unique social and economic environment. Thus, major stressors and their coping strategies differ greatly between citizens of Shanghai and those from other areas. This fact could introduce bias and decrease the generalizability to the current studies. Such points would be considered in future studies’ protocols.

## Conclusions

Conclusively, the current study provides some initial indication of high levels of perceived stress in the C-STRD residents and identifies the specific stressors that cause this high stress levels. Although there was a difference in perception of stress for workload and career future among different educational degree owners, low financial income is the major stressor among all C-STRD residents, which are consistent with the literatures [22, 37]. Unhealthy stress-reducing interventions are widely utilized by the C-STRD residents due to lack of a proper stress reduction program. Future research is recommended to seek for effective support service and proper guideline to ease the C-STRD residents’ stress.

## Supporting information

S1 Table The formal questionnair used in the current study. (PDF)

## References

[1] AlosaimiF, KazimS, AlmuflehA, AladwaniB, AlsubaieA. Prevalence of stress and its determinants among residents in Saudi Arabia. Saudi Med J. 2015;36(5):605–12. 10.15537/smj.2015.5.10814 25935183PMC4436759

[2] LourençãoL, MoscardiniA, SolerZ. Health and quality of life of medical residents. Rev Assoc Med Bras. 2010;56(1):81–91. 2033979210.1590/s0104-42302010000100021

[3] VeaseyS, RosenR, BarzanskyB, RosenI, OwensJ. Sleep loss and fatigue in residency training: a reappraisal. JAMA. 2002;288(9):1116–24. 1220408210.1001/jama.288.9.1116

[4] LockleyS, CroninJ, EvansE, CadeB, LeeC, LandriganC, et al Effect of reducing interns' weekly work hours on sleep and attentional failures. N Engl J Med. 2004;351(18):1829–37. 10.1056/NEJMoa041404 15509816

[5] ZisP, AnagnostopoulosF, SykiotiP. Burnout in medical residents: a study based on the job demands-resources model. ScientificWorldJournal. 2014;2014(673279).10.1155/2014/673279PMC423020525531003

[6] AnagnostopoulosF, DemeroutiE, SykiotiP, NiakasD, ZisP. Factors associated with mental health status of medical residents: a model-guided study. J Clin Psychol Med Settings. 2015;22(1):90–109. 10.1007/s10880-014-9415-2 25554496

[7] BittnerJ, KhanZ, BabuM, HamedO. Stress, burnout, and maladaptive coping: strategies for surgeon well-being. Bull Am Coll Surg. 2011;96(8):17–22. 22319907

[8] Anonymous. The impliment of standardized training for resident in Shanghai. Shanghai: Shanghai Municipal Health Bureau; 2010. http://www.smhb.gov.cn/wsj/n429/n432/n2354/n1546/u1ai81009.html.

[9] Anonymous. The management platform for Shanghai Standardized Training for Resident Doctor 2014. http://www.shrct.haoyisheng.com/.

[10] WaldmanS, DiezJ, AraziH, LinetzkyB, GuinjoanS, GrancelliH. Burnout, perceived stress, and depression among cardiology residents in Argentina. Acad Psychiatry. 2009;33(4):296–301. 10.1176/appi.ap.33.4.296 19690109

[11] AbutY, KitapciogluD, ErkalpK, ToprakN, BoztepeA, SivrikayaU, et al Job burnout in 159 anesthesiology trainees. Saudi J Anaesth. 2012;6(1):46–51. 10.4103/1658-354X.93059 22412777PMC3299115

[12] LebensohnP, DoddsS, BennR, BrooksA, BirchM, CookP, et al Resident wellness behaviors: relationship to stress, depression, and burnout. Fam Med. 2013;45(8):541–9. 24129866

[13] Al-SowyghZ. Academic distress, perceived stress and coping strategies among dental students in Saudi Arabia. Saudi Dent J. 2013;25(3):97–105. 2417931810.1016/j.sdentj.2013.05.002PMC3809483

[14] ZareS, GalankoJ, BehrnsK, KorudaM, BoyleL, FarleyD, et al Psychological well-being of surgery residents before the 80-hour work week: a multiinstitutional study. J Am Coll Surg. 2004;198(4):633–40. 10.1016/j.jamcollsurg.2003.10.006 15051017

[15] CostantinoC, AlbeggianiV, BonfanteM, MonteC, Lo CascioN, MazzuccoW. Cross-sectional study of the variability of work-related stress among post-graduate medical residents at the main University Polyclinic of Sicily. Med Lav. 2015;106(2):109–18. 25744311

[16] Walonick D. Survival Statistics StatPac Inc.; 2013.

[17] Anonymous. Developing a Survey Instrument.: Rutgers University; 2017. http://njaes.rutgers.edu/evaluation/resources/survey-instrument.asp.

[18] PhillipsJ, WilbanksD, SalinasD, DoberneckD. Educational Debt in the Context of Career Planning: A Qualitative Exploration of Medical Student Perceptions. Teach Learn Med. 2016;28(3):243–51. 10.1080/10401334.2016.1178116 27152504

[19] BelkićK, NedicO. Workplace stressors and lifestyle-related cancer risk factors among female physicians: assessment using the Occupational Stress Index. J Occup Health. 2007;49(1):61–71. 1731446810.1539/joh.49.61

[20] RichardsenA, BurkeR. Occupational stress and job satisfaction among physicians: sex differences. Soc Sci Med;33(10): 1991;33(10):1179–87. 176728810.1016/0277-9536(91)90234-4

[21] BovierP, PernegerT. Predictors of work satisfaction among physicians. Eur J Public Health. 2003;13(4):299–305. 1470331510.1093/eurpub/13.4.299

[22] AlhajjM, KhaderY, MuradA, CelebicA, HalboubE, MárquezJ, et al Perceived sources of stress amongst dental students: A multicountry study. Eur J Dent Educ. 2018: 10.1111/eje.12350 29607584

[23] CohenS, KamarckT, MermelsteinR. A global measure of perceived stress. J Health Soc Behav. 1983;24(4):385–96. 6668417

[24] ÖrücüM, DemirA. Psychometric evaluation of perceived stress scale for Turkish university students. Stress and Health. 2009;25(1):103–9.

[25] SmithK, RosenbergD, Timothy HaightG. An assessment of the psychometric properties of the perceived stress Scale-10 (PSS10) with business and accounting students. Accounting Perspectives. 2014;13(1):29–59.

[26] LeungD, LamT, ChanS. Three versions of Perceived Stress Scale: validation in a sample of Chinese cardiac patients who smoke. LeungDY, LamTH, ChanSS. BMC Public Health. 2010;10(513).10.1186/1471-2458-10-513PMC293964420735860

[27] McCueJ. The distress of internship. Causes and prevention. N Engl J Med 2 14; (7): 1985;312(7):449–52.396910710.1056/NEJM198502143120725

[28] CarverC, ScheierM, WeintraubJ. Assessing coping strategies: a theoretically based approach. J Pers Soc Psychol. 1989;56(2):267–83. 292662910.1037//0022-3514.56.2.267

[29] RadcliffeC, LesterH. Perceived stress during undergraduate medical training: a qualitative study. Med Educ. 2003;37(1):32–8. 1253511310.1046/j.1365-2923.2003.01405.x

[30] LloydC, GartrellN. A further assessment of medical school stress. J Med Educ. 1983;58(12):964–7. 664478010.1097/00001888-198312000-00008

[31] SalmonsP. Psychiatric illness in medical students. Br J Psychiatry. 1983;143:505–8. 664022110.1192/bjp.143.5.505

[32] ShanafeltT, BradleyK, WipfJ, BackA. Burnout and self-reported patient care in an internal medicine residency program. Ann Intern Med. 2002;136(5):358–67. 1187430810.7326/0003-4819-136-5-200203050-00008

[33] SmithJ, DennyW, WitzkeD. Emotional impairment in internal medicine house staff. Results of a national survey. JAMA. 1986;255(9):1155–8. 3945035

[34] ColfordJJ, McPheeS. The ravelled sleeve of care. Managing the stresses of residency training. JAMA. 1989;261(6):889–93. 2913386

[35] YaoD, WrightS. National survey of internal medicine residency program directors regarding problem residents. JAMA. 2000;284(9):1099–104. 1097468810.1001/jama.284.9.1099

[36] MurphyR, GrayS, SterlingG, ReevesK, DuCetteJ. A comparative study of professional student stress. J Dent Educ. 2009;73(3):328–37. 19289722

[37] HayesA, HooverJ, KarunanayakeC, UswakG. Perceived causes of stress among a group of western Canadian dental students. BMC Res Notes. 2017;10(1):714 10.1186/s13104-017-2979-9 29216910PMC5721618

[38] ZvauyaR, OyebodeF, DayE, ThomasC, JonesL. A comparison of stress levels, coping styles and psychological morbidity between graduate-entry and traditional undergraduate medical students during the first 2 years at a UK medical school. BMC Res Notes. 2017;10(1):93 10.1186/s13104-017-2395-1 28193287PMC5307866

[39] SandoverS, Jonas-DwyerD, MarrT. Graduate entry and undergraduate medical students' study approaches, stress levels and ways of coping: a five year longitudinal study. BMC Med Educ. 2015;24(15):5.10.1186/s12909-015-0284-7PMC431003825616440

[40] DyrbyeL, ThomasM, ShanafeltT. Systematic review of depression, anxiety, and other indicators of psychological distress among U.S. and Canadian medical students. Acad Med. 2006;81(4):354–73. 1656518810.1097/00001888-200604000-00009

[41] StewartS, LamT, BetsonC, WongC, WongA. A prospective analysis of stress and academic performance in the first two years of medical school. Med Educ. 1999;33(4):243–50. 1033675410.1046/j.1365-2923.1999.00294.x

[42] ParkK, KimD, KimS, YiY, JeongJ, ChaeJ, et al The relationships between empathy, stress and social support among medical students. Int J Med Educ. 2015;5(6):103–8.10.5116/ijme.55e6.0d44PMC456155326342190

[43] SherinaM, RampalL, NanesonN. Psychological Stress Among Undergraduate Medical Students. Med J Malaysia. 2003;59(2):207–11.15559171

[44] SaipanishR. Stress among medical students in a Thai medical school. Med Teach. 2003;25(5):502–6. 10.1080/0142159031000136716 14522672

[45] AbdulghaniH, AlKanhalA, MahmoudE, PonnamperumaG, AlfarisE. Stress and its effects on medical students: a cross-sectional study at a college of medicine in Saudi Arabia. J Health Popul Nutr. 2011;29(5):516–22. 2210675810.3329/jhpn.v29i5.8906PMC3225114

[46] WestC, ShanafeltT, KolarsJ. Quality of life, burnout, educational debt, and medical knowledge among internal medicine residents. JAMA. 2011;306(9):952–60. 10.1001/jama.2011.1247 21900135

[47] CollierV, McCueJ, MarkusA, SmithL. Stress in medical residency: status quo after a decade of reform? Ann Intern Med. 2002;136(5):384–90. 1187431110.7326/0003-4819-136-5-200203050-00011

[48] XuG, VeloskiJ. Debt and primary care physicians' career satisfaction. Acad Med. 1998;73(2):119 950838410.1097/00001888-199802000-00006

[49] 2011 Shanghai college graduates employment situation report [Internet]. China Bureau of Statitics. 2011. http://www.stats-sh.gov.cn/fxbg/201108/228620.html.

[50] Shanghai Household Final Consumption Expenditure [Internet]. China Bureau of Statitic. 2010. http://www.stats-sh.gov.cn/tjnj/nj11.htm?d1=2011tjnj/C0916.htm.

[51] WrennK, LorenzenB, JonesI, ZhouC, AronskyD. Factors affecting stress in emergency medicine residents while working in the ED. Am J Emerg Med. 2010;28(8):897–902. 10.1016/j.ajem.2009.05.001 20825921

[52] PhilibertI, FriedmannP, WilliamsW, ACGME Work Group on Resident Duty Hours. Accreditation Council for Graduate Medical Education. New requirements for resident duty hours. JAMA. 2002;288(9):1112–4. 1220408110.1001/jama.288.9.1112

[53] FletcherK, UnderwoodWr, DavisS, MangrulkarR, McMahonLJ, SaintS. Effects of work hour reduction on residents' lives: a systematic review. JAMA. 2005;294(9):1088–100. 10.1001/jama.294.9.1088 16145030

[54] FergusonC, KelloggK, HutterM, WarshawA. Effect of work-hour reforms on operative case volume of surgical residents. Curr Surg. 2005;62(5):535–8. 10.1016/j.cursur.2005.04.001 16125616

[55] SheltonJ, KummerowK, PhillipsS, ArbogastP, GriffinM, HolzmanM, et al Patient safety in the era of the 80-hour workweek. J Surg Educ. 2014;71(4):551–9. 10.1016/j.jsurg.2013.12.011 24776874PMC4852697

[56] BraselK, PierreA, WeigeltJ. Resident work hours: what they are really doing. Arch Surg. 2004;139(5):490–3. 10.1001/archsurg.139.5.490 15136348

[57] NadeemM, EffendiM, Hammad AtherM. Attrition in surgical residency programmes: Causes and effects. Arab J Urol. 2014;12(1):25–9. 10.1016/j.aju.2013.07.002 26019917PMC4434499

[58] SargentM, SotileW, SotileM, RubashH, BarrackR. Stress and coping among orthopaedic surgery residents and faculty. J Bone Joint Surg Am. 2004;86-A(7):1579–86. 1525211110.2106/00004623-200407000-00032

[59] RamirezA, GrahamJ, RichardsM, CullA, GregoryW. Mental health of hospital consultants: the effects of stress and satisfaction at work. Lancet. 1996;347(9003):724–8. 860200210.1016/s0140-6736(96)90077-x

